# Effects of adipose stem cell-conditioned medium on the migration of vascular endothelial cells, fibroblasts and keratinocytes

This article has been retracted.

**DOI:** 10.3892/etm.2013.887

**Published:** 2013-01-07

**Authors:** LI HU, JIAJIA ZHAO, JIARONG LIU, NIYA GONG, LILI CHEN

**Affiliations:** Department of Stomatology, Wuhan Union Hospital, Tongji Medical College, Huazhong University of Science and Technology, Wuhan, Hubei 430030, PR China

**Keywords:** adipose stem cell-conditioned medium, vascular endothelial cells, fibroblasts, keratinocytes, migration

## Abstract

Adipose stem cell-conditioned medium (ASC-CM) has been successfully used to treat multiple types of tissue and organ defects, including skin wounds both *in vitro* and *in vivo*. However, the mechanisms through which ASC-CM promotes wound healing remain unclear. We hypothesized that the wound healing effect of ASC-CM is mediated in part by the promotion of the migration of vascular endothelial cells, fibroblasts and keratinocytes, the three cell types essential for wound healing. We reported that ASC-CM stimulated the migration of these cells sequentially, and endothelial cells were the first cell type to respond to ASC-CM stimulation (4 h), followed by fibroblasts (12 h) and then keratinocytes (24 h). We also determined the optimal concentration of ASC-CM in stimulating these cells (50% dilution) in addition to the optimal time to intervene in order to maximize the wound healing activity of ASC-CM. Our data suggest an important role for ASC-CM in wound healing, possibly through the synthetic action of multiple adipose stem cell-derived cytokines that in turn promote cell migration. Thus, ASC-CM appears to have significant potential in wound healing applications.

## Introduction

Adipose-derived stem cells (ASCs) were first isolated by Zuk *et al*(1) in 2001 from adipose tissues. These cells are able to differentiate into multiple cell lineages including adipocytes, chondrocytes, osteoblasts, muscle cells, endothelial cells and neurocytes (2,3). The yield of mesenchymal stem cells from adipose tissues is much higher than that from bone marrow tissues, adipose tissues are more readily available and the derived stem cells are easier to culture, therefore ASCs are considered to be an ideal source for tissue engineering and have a significant application and research value (4–6). Previous studies have confirmed that adipose stem cell-conditioned medium (ASC-CM) has a marked promoting effect on wound healing (7).

In the skin wound healing process, keratinocytes, fibroblasts and vascular endothelial cells all play important roles and they are the first cell types activated by trauma. Activated cells participate in wound covering, granulation, scar tissue formation, wound remodeling and angiogenesis via a series of cellular activities, including migration and proliferation (8). It is known that the migration of these cells is a key step in the early wound healing process. However, the majority of previous studies have focused on the effect of ASCs on cell proliferation (9) rather than cell migration.

Our previous data have confirmed that ASCs promote the migration of these three types of cells *in vitro*. As ASCs are known to promote wound healing mainly through a paracrine mechanism, it is plausible that ASCs may exert their effect by secreting cytokines and growth factors that act on neighboring cells to repair the damaged tissues (10–11). In terms of the potential clinical application of ASCs, a few issues have to be resolved such as the selection of an appropriate scaffold (12) and the integration of various cytokines into other tissues. However, ASC-CM has distinct advantages, including that it may be applied locally or via intravenous injection. More importantly, the levels of major cytokines in the ASC-CM may be precisely quantitated. Thus, ASC-CM may be more feasible and practical to use in wound healing than ASCs themselves. However, it is unknown whether ASC-CM influences cell migration, and if so, what the optimal concentrations and intervention times for different cells are. We therefore investigated the effect of ASC-CM on the migration of human keratinocytes, fibroblasts and vascular endothelial cells.

## Materials and methods

### Isolation and culture of primary human keratinocytes and fibroblasts

Human foreskins were obtained from donors (16–30 years old) undergoing circumcision after giving their informed consent. All procedures were approved by the ethics committee of Wuhan Union Hospital (Wuhan, China). The foreskins were washed several times with sterile phosphate-buffered saline (Thermo Scientific Hyclone, Rockford, IL, USA) and digested as described by Häkkinen *et al*(13) for isolation of keratinocytes and fibroblasts. The EA.hy926 cell line was used as an alternative for human umbilical vein endothelial cells (HUVECs). These cells were cultured at 37°C in 5.0% CO_2_. The media were replaced every 2–3 days.

### Isolation, characterization and multi-differentiation assay of human adipose-derived stem cells (ASCs)

Human subcutaneous adipose tissues were obtained from female patients (18–35 years old) undergoing lipoaspiration surgery after informed consent was obtained from the patient and approval provided by the ethics committee of Wuhan Union Hospital. The procedures described by Bunnell *et al*(2) were followed. Cells of passages 3–7 were used in the present study. Surface markers CD13, CD14, CD44, CD90, CD105 and CD34 were detected using a fluorescence-activated cell sorter. Following the differentiation of ASCs in various directions, such as adipogenesis and osteogenesis, the adipogenic lineage was detected by Oil Red O (Sigma-Aldrich, St. Louis, MO, USA) staining and the osteogenic lineage was detected by Alizarin red (Sigma-Aldrich) staining.

### Preparation of ASC-CM and protein microarray analysis

ASCs were cultured in DMEM/F-12 containing 10% fetal bovine serum until the cells reached 80% confluence. The culture medium was then replaced by serum-free DMEM/F-12 and incubated for an additional 48 h. The conditioned medium was collected, centrifuged at 165 g for 5 min and filtered through a 0.22-*μ*m syringe filter. The ASC-CM was stored at −20°C and 5 ml medium was used for protein array analysis with the RayBio^®^ Biotin Label-based Human Antibody Array I (AAH-BLM-1-2; RayBiotech, Norcross, GA, USA) which contains antibodies for 507 human proteins.

### Migration assays

The effect of ASC-CM on cell migration was determined using a modified Boyden Chamber assay. Briefly, 1×10^5^ HUVECs, fibroblasts or keratinocytes were seeded into the upper chambers, with 300 *μ*l culture medium in the upper chambers and 600 *μ*l culture medium in the lower chambers. After the cells adhered to the bottom of the upper chambers, the medium in the upper chambers was replaced by serum-free DMEM/F-12. The medium in the lower chambers was replaced with medium containing different concentrations of ASC-CM (0, 10, 25, 50, 75 and 100%). In our preliminary studies, we observed that HUVECs clearly migrated within a few hours. However, fibroblasts began to migrate after ten hours, while keratinocytes began to migrate within one or two days. Therefore, we chose to evaluate HUVEC migration within the period of 4–20 h, fibroblasts at 12–36 h and keratinocytes at 24–72 h. Cells on the upper surface of the inserts were removed using a cotton swab and those that had migrated through the filter were stained with crystal violet. Cells in 16 microscopic fields at ×200 magnification were counted. The experiments were performed in triplicate.

### Statistical analysis

The values are expressed as mean ± standard deviation. Comparisons between two groups were analyzed by Student’s t-test and comparisons among more than two groups were obtained by ANOVA. P<0.05 was considered to indicate a statistically significant result. The analyses were performed using SPSS 16.0 (SPSS Inc., Chicago, IL, USA).

## Results

### Morphology, flow cytometry and multi-differentiation analysis

HUVECs were flat and polygonal-shaped, arranged in short spindles or a cobblestone morphology (Fig. 1A). The primary skin keratinocytes also had cobblestone morphology, a characteristic of epithelial cells in an undifferentiated stage (Fig. 1B). The primary fibroblasts were spindle-shaped and distributed in a radial or swirl shape (Fig. 1C). In the primary and first passage, ASCs proliferated slowly and generated a homogeneous population of flat and fibroblast-like cells after 3 passages (Fig. 2A–D). Flow cytometry showed that the ASCs were positive for CD13 (99.49%), CD44 (92.13%), CD90 (97.78%) and CD105 (96.82%) but negative for CD14 (1.14%) and CD34 (2.71%; Fig. 2E). In order to determine the multipotency of the ASCs, the cells were cultured in adipogenic and osteogenic differentiation medium and the multi-differentiation potential was confirmed by lipid vacuoles positive for Oil Red O staining (Fig. 2F) and colonies positive for Alizarin red staining (Fig. 2G).

### Protein microarray analysis of ASC-CM

The amounts of cytokines secreted by ASCs into the medium were analyzed by protein microarrays of ASC-CM. As shown in Fig. 2H, a total of 268 cytokines had a signal that exceeded 300 times that of the background following normalization against the internal control (IC). Among them were 57 common cytokines that have known properties that have the potential to influence cell migration (Table I).

### Determination of the optimal concentration of ASC-CM to promote the migration of HUVECs, fibroblasts and keratinocytes

In order to investigate whether ASC-CM impacts the migration of HUVECs, fibroblasts and keratinocytes and to determine the optimal ASC-CM concentration, we performed a dose-response experiment, in which serially diluted ASC-CM (0, 10, 25, 50, 75 and 100%) was added to the lower chambers and its ability to induce cell migration was measured. The stained cells are shown in Fig. 1 [(D) HUVECs, (E) keratinocytes, (F) fibroblasts]. Fig. 3 shows that the migratory effects of 50% ASC-CM on HUVEC, fibroblast and keratinocyte migration were significantly higher than those of either lower concentrations (0, 10 and 25%) or higher concentrations (75 and 100%; P<0.05; Fig. 3A–C). The average numbers of HUVECs, fibroblasts and keratinocytes that migrated to the other side of the chamber in the 50% ASC-CM treated group were 122.69±22.02, 90.88±16.52 and 46.00±10.59, respectively.

### Migration assay of HUVECs, fibroblasts and keratinocytes stimulated by 50% ASC-CM for different time periods

To further characterize the effect of ASC-CM on different types of cells and determine the cell types most sensitive in responding to ASC-CM, we examined the responsiveness of HUVECs, fibroblasts and keratinocytes toward 50% ASC-CM for different time periods. The results shown in Fig. 3D–F indicate that the migration of HUVECs occurred the fastest. ASC-CM-stimulated HUVEC migration started within 4 h and peaked at 12 h. Fibroblasts were the second fastest to respond. Fibroblasts started to migrate at 12 h and reached a maximum at 24 h. Keratinocytes appeared to be the slowest to respond to ASC-CM stimulation with the first appearance of migration at 24 h and reaching a maximum at 60 h (P<0.05; Fig. 3D–F, Fig. 4). The net increase in the number of migrated cells was greatest in the period of 4–8 h for HUVECs and 18–24 h for fibroblasts, while keratinocytes kept a constant rate of migration over the time period of this study (Fig. 4 and Table II).

## Discussion

Epithelial keratinocytes, dermal fibroblasts and local vascular endothelial cells play significant roles in the skin wound healing process. Previous studies have reported that ASCs are able to accelerate wound healing, possibly through a paracrine mechanism. ASC-CM contains a number of cytokines secreted by ASCs. The effect of these cytokines on cell proliferation has been extensively studied. However, it is less clear whether ASC-CM also influences cell migration and if so, whether it is dose-dependent and what is the optimal intervention timing for different cells. We therefore addressed these unanswered questions in the current study and the results reported in this paper provide a more comprehensive understanding of the effect of ASC-derived cytokines on wound healing.

Previous studies have shown that cytokines including VEGF, bFGF, Ang-1, Ang-2, CDK-5, CD44 and PECAM-A (14–17) are important in promoting the migration of endothelial cells. Kanazawa *et al*(18) also reported that bFGF may activate RhoA, Rac1, PI3-kinase and JNK in cultured fibroblasts, and promote fibroblast migration. In addition, Maheshwari *et al*(19) observed that epidermal growth factor (EGF) and fibronectin had a synergistic effect on fibroblast migration. Concerning the migration of keratinocytes, Bae *et al*(20) reported that keratinocytes could be induced by TGF-β to express the extracellular matrix protein βig-h3 that supported keratinocyte migration by interacting with α3β1 integrin. The results of the protein microarray analysis in the current study demonstrated that ASCs are able to secret multiple cytokines including VEGF, HGF, TGF-β, EGF, FGF, SDF-1 and Ang-1. In addition, flow cytometry revealed high expression levels of CD44 on ASCs. These results suggest an important role for ASCs in wound healing, likely through the secretion of multiple cytokines that in turn promote cell migration.

In particular we studied the effect of ASC-CM on the migration of endothelial cells, fibroblasts and keratinocytes. The results showed that cell migration increased with increasing concentrations of ASC-CM and reached a maximum with 50% of ASC-CM (Fig. 3). Further increases of ASC-CM concentration did not result in any further increase in cell migration but instead diminished cell migration. The low migratory activity at low ASC-CM concentration is likely to be due to the low concentration of cytokines. However, it is currently unknown why a high concentration of ASC-CM is inhibitory. One possible reason is the existence of inhibitory factors in the conditioned medium. The optimal dose of stimulatory and inhibitory cytokines may be different. At the same concentration of ASC-CM, HUVECs were the first to migrate (Fig. 4), followed by fibroblasts and then keratinocytes. These results are consistent with a recent study which suggested that during the tissue remodeling stage of wound healing, dermal fibroblasts along with microvascular endothelial cells may migrate into the wound area prior to keratinocytes (21). Under the optimal concentration of ASC-CM (50%), the increase of HUVEC migration was greatest in the period of 4–8 h and that of fibroblasts was greatest in the period of 18–24 h, while the speed of keratinocyte migration remained constant over the 72 h. Therefore, the optimal intervention timing for vascular endothelial cell migration and fibroblast migration were within 8 and 24 h, respectively. The intervention point for keratinocyte migration was not time-sensitive. Notably these results were generated from *in vitro* studies. Wound healing *in vivo* is a much more complex process, so further *in vivo* studies are required to fully understand the effect of ASC-CM on the migration of different cells in a more physiologically relevant setting.

## Figures and Tables

**Figure 1.** (A) Human umbilical vein endothelial cells (HUVECs), (B) keratinocytes and (C) fibroblasts from skin, ×100 magnification. Cells stained with crystal violet after migration, (D) HUVECs, (E) keratinocytes and (F) fibroblasts, ×200 magnification.

**Figure 2.** Isolation and culture of human adipose-derived stem cells (hASCs) *in vitro* [(A) P0 (B) P1 (C) P2 (D) P3, ×100 magnification]. (Ea-d) Flow cytometry performed on the hASCs in the 3rd passage showed that isolated hASCs positively expressed CD13, CD44, CD90, CD105 and negatively expressed CD14, CD34. (F) Adipogenic differentiated ASCs were positively stained by Oil Red O. (G) Osteogenic differentiated adipose-derived stem cells (ASCs) were positively stained by Alizarin red. (H) Protein microarray analysis of ASC-CM. ASC-CM, ASC-conditioned medium. P0, primary ASCs; P1, passage 1; P2, passage 2; P3, passage 3.

**Figure 3.** The effect of different concentrations of adipose stem cell-conditioned medium (ASC-CM) on migration of (A) human umbilical vein endothelial cells (HUVECs), (B) fibroblasts and (C) keratinocytes. The migratory effects of 50% ASC-CM were significantly greater than those of either lower concentrations (0, 10 and 25%) or higher concentrations (75 and 100%). Migration assay of (D) HUVECs, (E) fibroblasts and (F) keratinocytes stimulated by 50% ASC-CM at different time periods. Results showed that HUVEC migration started at 4 h, and peaked at 12 h. Fibroblasts started to migrate at 12 h and reached a maximum in 24 h. Keratinocytes appeared to be the slowest to respond to ASC-CM stimulation. Control, 0% ASC-CM; ^*^P<0.05.

**Figure 4.** Comparison of the migration of human umbilical vein endothelial cells (HUVECs), fibroblasts and keratinocytes stimulated by 50% adipose stem cell-conditioned medium (ASC-CM). Results showed 50% ASC-CM had a clear effect on cell migration, particularly on HUVEC and fibroblast migration, but the effect on keratinocyte migration was less marked, with 0% ASC-CM as the control.

**Table I.** Common cytokines whose internal control normalization without background exceeded 300 in ASC-CM.

Cytokine	Internal control
EDA-A2	10,056.00
IGFBP-7	6,651.00
TSP	4,544.50
RTIMP-1	3,221.50
SPARC	2,607.00
GDF3	1,400.50
NRG3	1,328.50
HCR/CRAM-A/B	1,261.00
MSP α chain	1,253.50
MMP-20	1,085.00
TGF-β5	839.00
IL-22	811.50
FGF-11	800.50
CNTF	704.00
FGF R4	697.00
Angiopoietin-like 1	627.50
MMP-7	566.50
Insulin R	541.00
Endothelin	540.00
CTGF/CCN2	524.00
CCR4	523.50
CXCR2/IL-8	503.50
MMP-1	501.00
BMP-8	493.00
IGF-II	486.00
BMP-5	476.50
VEGF R2 (KDR)	469.50
MMP-15	467.50
G-CSF R/CD114	464.00
HB-EGF	458.00
PF4/CXCL4	456.00
MMP-3	455.00
CCR5	450.50
CXCR6	450.50
IGF-ISR	449.50
HGF	444.00
FGF-16	425.00
Angiopoietin-like 2	419.50
MMP-13	416.50
FGF-10/KGF-2	413.00
FGF-9	410.50
BMP-4	405.50
TGF-β2	402.50
SDF-1/CXCL12	400.00
VEGF R3	396.00
VEGF-D	395.00
FGF Basic	389.50
MMP-8	371.50
PDGF-AA	363.50
Angiopoietin-like factor	361.50
VEGF	360.50
MMP-2	359.00
Angiopoietin-1	352.50
Angiopoietin-4	342.50
IL-1β	333.00
PDGF-BB	312.50
TNF-β	309.00

ASC-CM, adipose stem cell-conditioned medium.

**Table II.** Effects of 50% ASC-CM on the migration of HUVECs, fibroblasts and keratinocytes over different time periods.

		Migration cells/field			
Cell	Time (h)	50% ASC-CM	Control	M1	M2
HUVEC	4	80.63±15.82	33.63±14.80	47.00	-
	8	122.69±22.02	43.13±21.86	79.56	32.56
	12	151.69±57.74	60.25±14.99	91.44	11.88
	16	141.56±29.14	58.38±11.54	83.19	−8.25
	20	130.19±22.36	49.19±14.57	81.00	−2.19
Fibroblast	12	62.19±27.46	23.19±10.42	39.00	-
	18	90.88±16.52	26.94±13.40	63.94	24.94
	24	136.69±10.20	44.81±11.31	91.88	27.94
	30	125.44±23.55	51.13±9.27	74.31	−17.56
	36	118.94±21.66	48.81±7.33	70.13	−4.19
Keratinocyte	24	32.94±12.17	18.00±8.70	14.94	-
	36	39.56±13.49	21.25±9.50	18.31	3.38
	48	46.00±10.59	24.25±11.13	21.75	3.44
	60	54.44±11.55	29.50±10.52	24.94	3.19
	72	53.81±11.73	32.13±10.59	21.69	−3.25

At each time point, cells stimulated by 50% ASC-CM migrated more than control cells. The net increase of migrated cells was greatest between 4–8 h for HUVECs and 18–24 h for fibroblasts, while keratinocytes demonstrated a constant migration over the entire time period. (M1=M_(50% ASC−CM)_−M_(control)_, M2=Mn−M_n−1_). ASC-CM, adipose stem cell-conditioned medium; HUVEC, human umbilical vein endothelial cell.
